# S100A9 gene silencing inhibits the release of pro‐inflammatory cytokines by blocking the IL‐17 signalling pathway in mice with acute pancreatitis

**DOI:** 10.1111/jcmm.13532

**Published:** 2018-02-14

**Authors:** Dong‐Mei Wu, Shan Wang, Min Shen, Yong‐Jian Wang, Bo Zhang, Zi‐Qi Wu, Jun Lu, Yuan‐Lin Zheng

**Affiliations:** ^1^ Key Laboratory for Biotechnology on Medicinal Plants of Jiangsu Province School of Life Science Jiangsu Normal University Xuzhou China; ^2^ College of Health Sciences Jiangsu Normal University Xuzhou China; ^3^ Department of General Surgery The First Affiliated Hospital of Fujian Medical University Fuzhou China

**Keywords:** acute pancreatitis, interleukin‐17 signalling pathway, pro‐inflammatory cytokine, S100A9

## Abstract

The study aimed to investigate whether S100A9 gene silencing mediating the IL‐17 pathway affected the release of pro‐inflammatory cytokines in acute pancreatitis (AP). Kunming mice were assigned to the normal, AP, AP + negative control (NC), AP + shRNA, AP + IgG and AP + anti IL‐17 groups. ELISA was applied to measure expressions of AMY, LDH, CRP, TNF‐α, IL‐6 and IL‐8. The cells were distributed into the control, blank, NC, shRNA1 and shRNA2 groups. MTT assay, flow cytometry, RT‐qPCR and Western blotting were used to evaluate cell proliferation, cell cycle and apoptosis, and expressions of S100A9, TLR4, RAGE, IL‐17, HMGB1 and S100A12 in tissues and cells. Compared with the normal group, the AP group displayed increased expressions of AMY, LDH, CRP, TNFα, IL‐6, IL‐8, S100A9, TLR4, RAGE, IL‐17, HMGB1 and S100A12. The AP + shRNA and AP + anti IL‐17 groups exhibited an opposite trend. The in vivo results: Compare with the control group, the blank, NC, shRNA1 and shRNA2 groups demonstrated increased expressions of S100A9, TLR4, RAGE, IL‐17, HMGB1 and S100A12, as well as cell apoptosis and cells at the G1 phase, with reduced proliferation. Compared with the blank and NC groups, the shRNA1 and shRNA2 groups had declined expressions of S100A9, TLR4, RAGE, IL‐17, HMGB1 and S100A12, as well as cell apoptosis and cells at the G1 phase, with elevated proliferation. The results indicated that S100A9 gene silencing suppressed the release of pro‐inflammatory cytokines through blocking of the IL‐17 pathway in AP.

## 1 INTRODUCTION

Acute pancreatitis (AP) relates to an acute inflammatory progression, by which the pancreas elicits a systemic inflammatory response.^1^ It is widely accepted that AP refers to a dynamic evolving situation, with fluctuations in severity during the development of the disease.^2^ Severe acute pancreatitis (SAP) represents the most serious type of AP largely due to the fact comes with particularly high rates of morbidity and mortality.^3^ Biliary pathology and alcohol misuse typify the most typical patterns of AP aetiology, accounting for 40% and 22% of all cases of the condition, respectively. Furthermore, other risk factors associated with the condition include trauma, hypercholesterolaemia, iatrogenic procedures and other idiopathic causes.^4^ It is estimated that approximately 30% of all AP patients will be subject to severe attacks, which is indicative of a high mortality rate.^5^ Owing to both the high mortality rate and exorbitant medical costs associated with the treatment of the more severe cases of AP, treatment of AP remains a critical challenge to the field of gastroenterology.^6^ Schenckenburger et al demonstrated the roles of S100 calcium‐binding protein A9 (S100A9) in inflammatory cell infiltration and in cell‐cell contact regulation.^7^ S100A9, which is commonly referred to as myeloid‐related protein‐14 (MRP14), is a primary member of the S100 family of proteins and has been linked to acute and chronic inflammatory conditions.^8^ Furthermore, elevated levels of S100A8/A9 have been detected in a variety of inflammatory diseases, such as rheumatoid arthritis and inflammatory bowel disease.^9^ During this study, we aimed to elucidate the mechanisms involved with S100A9 and its role in AP.

When combined with S100A8, S100A9 constitutes the heterodimeric protein calprotectin (S100A8/9), which is expressed in nearly all cells, tissues and fluids in the human body.^10^ A recent study explored the relationship between pancreatic cancer, S100A9/A8 and transforming growth factor beta 1 (TGFβ1) concluded that the overexpression of S100A9/A8 by infiltrating inflammatory cells and the expressions is related to TGFβ1 in pancreatic ductal adenocarcinoma (PDAC).^11^ Interleukin‐17 (IL‐17), a pro‐inflammatory cytokine mainly produced by T‐helper 17 (Th 17) cells, has been reported to play a crucial role in the development of an effective immune response.^12^, ^13^ Liu et al reported that IL‐17 played a pivotal role in the pathogenesis of numerous inflammatory diseases in the central nervous system (CNS), such as multiple sclerosis and stoke,^14^ whereas Dai et al suggested that serum IL‐17 was an early prognostic biomarker of severe acute pancreatitis in patients receiving continuous blood purification.^15^ However, few studies have appeared to place an emphasis on the effects of S100A9 and the release of pro‐inflammatory cytokines through the IL‐17 signalling pathway in AP. Hence, during this study, we aimed to explore the roles of S100A9 in the release of pro‐inflammatory cytokines via the IL‐17 signalling pathway in a mouse model of AP.

## 2 MATERIALS AND METHODS

### 2.1 Ethics statement

All animal use and experimental procedures were performed in accordance with the Declaration of Helsinki,^16^ as well as in agreement with the Experimental Animal Ethics Committee of Key Laboratory for Biotechnology on Medicinal Plants of Jiangsu Province, School of Life Science, Jiangsu Normal University.

### 2.2 Establishment of AP mouse model

A total of 90 healthy male Kunming (KM) mice were raised under a specific pathogen animal (SPF) environment (23°C room temperature, 65% relative humidity and 12/12 hours light/dark cycle), with free access to water and food deprivation a minimum of 12 hours. The mice were then divided into 6 groups (15 mice each group), namely a normal (intraperitoneally injected with the same volume of sterile normal saline 6 times, once/h), a AP group (intraperitoneally injected with 20% L‐arginine [L‐Arg] [200 mg/100 g] [S3174, Selleck Chemicals Co. Ltd., Shanghai, China] 6 times, once/h), a AP + negative control (NC) group (injected with 200 μL 5 × 10^9^ TU/mL shRNA‐NC lentivirus by tail vein before intraperitoneal injection with 20% L‐Arg), a AP + shRNA group (injected with 200 μL 5 × 10^9^ TU/mL shRNA‐S100A9 lentivirus by tail vein before intraperitoneal injection with 20% L‐Arg), a AP + IgG group (intraperitoneally injected with IgG isotype control protein every 48 hours [4 times, 100 μg per mouse] [Tianjin Sungene Biotech Co., Ltd., Tianjin, China]) and a AP + anti IL‐17 group (intraperitoneally injected with IL‐17 monoclonal antibody every 48 hours [4 times, 100 μg per mouse] [Tianjin Sungene Biotech Co., Ltd., Tianjin, China]).^17^ When the mice exhibited a reduction in foraging activity, a tendency to huddle, loose fur, distended abdomens and frequent urination, post‐model establishment, the model was then considered to be successful.^18^ Twenty‐four hours post‐model establishment, a tail bleeding procedure was performed. The mice were executed, and the serum was separated and stored in a refrigerator at −20°C. One part of the extracted pancreatic tissues was fixed, embedded and sectioned for immunohistochemistry (IHC) and haematoxylin‐eosin (HE) staining, whereas the other part was used for reverse transcription quantitative polymerase chain reaction (RT‐qPCR) and Western blotting purposes.

### 2.3 Immunohistochemistry (IHC)

Immunohistochemistry was performed in accordance with the instructions of the SP‐9001 Kit (Beijing Nobleryder Technology Co. Ltd., Beijing, China). The paraffin‐embedded pancreatic tissue blocks obtained from the mice of the normal and AP groups were placed at room temperature for 30 minutes. The tissues were then fixed with acetone at 4°C for 10 minutes, dewaxed and rehydrated. After the tissues were washed 3 times with phosphate‐buffered saline (PBS) (5 minutes per wash), 3% H_2_O_2_ was used to exhaust the endogenous peroxidase activity for 5‐10 minutes. The blocks were then washed 3 times with distilled water (3 minutes per wash) and immersed twice in PBS (5 minutes each time). After that, the tissues were blocked finally in a working solution comprised of 5% normal goat serum (C1771, Beijing Applygen Technology Co., Ltd, Beijing, China). After incubation at 37°C for 10‐15 minutes, the tissue blocks were sliced into sections of approximately 5 μm, which were flattened and baked at 70°C for 1 hour, followed by slicing and an additional round of baking at 60°C for 5. Next, the sections were incubated with rabbit anti‐S100A9 antibody (ab92507, Abcam Inc., Cambridge, MA, USA) and IL‐17 (ab79056, Abcam Inc., Cambridge, MA, USA) at 4°C overnight. The sections were then placed at room temperature for 30 minutes, washed 3 times with PBS (5 minutes each time) and incubated with a corresponding biotinylated goat anti‐rabbit IgG secondary antibody (ab150077, Abcam Inc, Cambridge, MA, USA) at 37°C for 1 hour. After an additional 3 washes with PBS (5 minutes each time), the sections were incubated with horseradish peroxidase (HRP) (0343‐10000U, Beijing Imun Biotechnology Co., Ltd., Beijing, China) labelled streptavidin working solution at 37°C for 1 hour, followed by 3 further PBS washes (5 minutes each time). A 3,3′‐diaminobenzidine (DAB, ST033, Guangzhou Whiga Technology Co., Ltd., Guangzhou, Guangdong, China) was used for colour development for a period of 3‐10 minutes, and the samples were washed with double‐distilled water (DDW) for 10 minutes after the reaction had been stopped. The sections were then counterstained with haematoxylin (Shanghai Fusheng Industrial Co., Ltd., Shanghai, China) for 1 minute and soaked in 1% hydrochloric acid‐ethanol mixtures for 10 seconds. After washing with running water, the tissues were stained to turn blue for 10 seconds using 1% ammonia. Next, the samples were dehydrated with graded ethanol, permeabilized with xylene and mounted by neutral balsam. PBS was regarded as the NC during the replacement of the primary antibody. The experiment was repeated 3 times. The scores of staining intensity and cell rate of positive expression were calculated using the OlymPusDp70 image acquisition analyser. The scale of staining intensity was as follows: 0, no staining; 1, weak staining; 2, moderate staining; 3, strong staining. The criteria for the cell rate of positive expression were as follows: 0, <1%; 1, <10%; 2, <50%; 3, <80%; 4, >80%; The final score was calculated based on staining intensity and cell rate of positive expression: 0‐2, negative (−); 3‐5, positive (+); 6‐7, strongly positive (++).

### 2.4 Haematoxylin‐eosin (HE) staining

The pancreatic tissues were extracted from the executed mice and immediately fixed in 4% paraformaldehyde. The fixed tissues were washed with running water, 24 hours later, dehydrated conventionally once for 1 minute, permeabilized twice in xylene (5 minutes each time), dipped in wax and cooled on the cooling stage of the paraffin embedding station. The embedded blocks were sliced at a thickness of 5 μm, which were flattened, baked at 70°C for 1 hour and then further baked again at 60°C for 5 hours. The paraffin‐embedded sections were deparaffinized and rehydrated, stained with haematoxylin for 10 minutes at room temperature and washed with running water for a duration of 30‐60 seconds. Next, the tissue blocks were differentiated with 1% hydrochloric acid‐ethanol mixtures, washed with running water for 5 minutes and stained with eosin (0001‐H, Beijing Xinhua Lvyuan Science & Technology Co., Ltd, Beijing, China) at room temperature for 1 minute. The samples were then dehydrated with gradient ethanol (70%, 80%, 90%, 95% and 100%) for 1 minute, respectively, immersed in carbolic acid xylene and permeabilized twice in xylene I and II (GD‐RY1215‐12, Shanghai Guduo Biotechnology Co., Ltd., Shanghai, China), respectively (1 minute each time). Finally, a sealing process was performed using neutral balsam in the fume hood. Images were obtained by means of photography using a Zeiss fluorescence microscope (PrimoStar iLED, Bio‐Research (Beijing) Scientific Co., Ltd., Beijing, China), whereas the pathological changes among the pancreatic tissues were recorded.

### 2.5 Enzyme‐linked immunosorbent assay (ELISA)

Serum from mice in the normal and AP groups was collected. An ELISA Kit (YQ, Beijing Imun Biotechnology Co., Ltd., Beijing, China) was used to detect the amylase serum levels (AMY, JK‐EA01139), lactate dehydrogenase (LDH, JKSJ‐1983), c‐reactive protein (CRP, JK‐(a)‐1623), tumour necrosis factor α (TNFα, JK‐EA01383), interleukin‐6 (IL‐6, JKSJ‐2176) and interleukin‐8 (IL‐8, JKSJ‐1931) (all were purchased from Shanghai Jingkang Bioengineering Co., Ltd., Shanghai, China). The known antigen was diluted to 1‐10 μg/mL with a carbonate coating buffer (pH 9.6) and seeded into a 96‐well plate, followed by incubation at 4°C overnight with 0.1 mL diluent supplemented for each well. The solution in the well was removed the next day. Following 3 washes with a washing buffer (3 minutes each time), the well was supplemented with 0.1 mL sample supernatant, incubated at 37°C for 1 hour and washed again. Meanwhile, the blank, negative and positive control wells were set in the corresponding reaction wells. Next, the wells were added with 0.1 mL of enzyme‐labelled antibody (Abcam Inc, Cambridge, MA, USA) and incubated at 37°C for 35‐40 minutes, followed by washing with washing buffer and a final round of washing with ddH2O. Freshly prepared 0.1 mL substrate solution of tetramethyl benzidine (TMB, EL0001, Huzhou InnoReagents Co., Ltd., Huzhou, Zhejiang, China) was supplemented into each well for chromogen at 37°C for 10‐30 minutes. After 0.05 mL of 2 mol/L sulphuric acid was supplemented into each well, the optical density (OD) value was measured at 450 nm using a microplate reader (BS‐1101; Nanjing Detie Experimental Equipment Co., Ltd., Nanjing, Jiangsu, China). The OD value was measured when the value of the blank control well was zero.

### 2.6 Reverse transcription quantitative polymerase chain reaction (RT‐qPCR)

Pancreatic tissues (5 × 5 ×  5 mm^3^) were extracted from mice in of the AP and normal groups and then placed in 1 mL TRIZOL Kit (15596‐018, Beijing Solarbio Science & Technology Co., Ltd., Beijing, China). The tissues were homogenized for 2 minutes in an ice bath and centrifuged (10000 g rpm, 5 minutes), and the precipitate was discarded accordingly. Next, 200 μL chloroform was added to the tissues, mixed and placed at room temperature for 15 minutes at 4°C, followed by centrifugation at 12 000 rpm for 15 minutes. The extracted aqueous phase in the upper layer was mixed with 0.5 mL isopropyl alcohol, placed at room temperature for 10‐30 minutes and centrifuged at 4°C at 12 000 rpm for 10 minutes. Following the discarding of the supernatant, 1 mL 75% ethanol was added to the RNA precipitation in the bottom of tube, diluted with 20 μL diethyl pyrocarbonate (DEPC) and shaken gently to suspend the precipitate. After centrifugation at 4°C (8000 rpm, 5 minutes) to discard the supernatant, the samples were dried by means of airing at room temperature and in certain cases, vacuumed for 5‐10 minutes. DEPC (20 μL) was used to dissolve the precipitation, followed by determination of RNA concentration. The primer sequences were synthesized by Takara (Takara Biotechnology Co., Ltd., Dalian, China; Table 1), and then, reverse transcription was performed using the Reverse Transcription Kit (Beijing Transgen Biotechnology Co., Ltd., Beijing, China) in accordance with the manufacturer's instructions. The reaction conditions were as follows: 42°C for 30‐50 minutes (reverse transcription) and 85°C for 5 seconds (enzyme deactivation). Reversely transcribed cDNA was diluted to 50 ng/μL (adding 2 μL each time), whereas the amplification system was 25 μL. The fluorescence quantitative PCR instrument (ViiA 7, Da An Gene Co., Ltd. of Sun Yat‐Sen University, Guangdong, China) were adopted. The reaction condition of PCR included 40 cycles of pre‐denaturation at 95°C for 10 minutes, denaturation at 95°C for 5 seconds, annealing and elongation at 60°C for 30 seconds. The 2 μg RNA was used as template and glyceraldehyde‐3‐phosphate dehydrogenase (GAPDH) as the internal control. The 2^−ΔΔCT^ 19 method was used to calculate the relative mRNA expressions of target genes (S100A9, IL‐17, high‐mobility group box 1 protein (HMGB1) and S100A12):▵▵Ct = ▵Ct_AP group_ − ▵Ct_normal group_, ▵Ct = Ct_(target gene)_ − Ct_(internal control)_. Total RNA was extracted from the pancreas of the mice post‐transfection and incubated for 48 h. The same procedure was conducted for all cell experiments.

**Table 1:** Primer sequences for RT‐qPCR

Gene	Primer sequence (5′‐3′)
S100A9	F: TCATCGACCCTTCCATCAA
	R: GATCAACTTTGCCATCAGCA
IL‐17	F: GGTCAACCTCAAAGTCTTTAACTC
	R: TTAAAAATGCAAGTAAGTTTGCTG
HMGB1	F: GGGTCACATGGATTATTAGTG
	R: CAGGGCATGTGGACAAAAG
S100A12	F: CTTCCACCAATACTCAGTTCGG
	R: GCAATGGCTACCAGGGATATG
TLR 4	F: AGTGGGTCAAGGAACAGAAGCA R: CTTTACCAGCTCATTTCTCA CC
RAGE	F: AACACAGCCCCCATCCAA R: GCTCAACCAACAGCTGAATGC
GAPDH	F: AATGGGCAGCCGTTAGGAAA
	R: GCGCCCAATACGACCAAATC

F, forward; R, reverse; S100A9, S100 calcium‐binding protein A9; IL‐17, interleukin‐17; HMGB1, high‐mobility group box 1 protein; S100A12, calgranulin C; TLR4, toll‐like receptor 4; RAGE, receptor for advanced glycation end products; GAPDH, glyceraldehyde‐3‐phosphate dehydrogenase; RT‐qPCR, reverse transcription quantitative polymerase chain reaction.

### 2.7 Western blotting

After weighing, the cooled pancreatic tissues from each group were placed in a glass grinder containing 1 mL ice‐cold normal saline. After homogenization in an ice bath, the tissues were centrifuged (12 000 rpm/min) at 4°C for 20 minutes, and the supernatant was discarded. Next, 1 ml of lysates (including 50 mmol/LT ris, 150 mmol/L NaCl, 5 mmol/L ethylene diamine tetraacetic acid (EDTA), 0.1% sodium dodecyl sulphate (SDS), 1% NP‐40, 5 g/mL Aprotinin and 2 mmol/L phenylmethanesulfonyl fluoride (PMSF)) was added to the tissues and triturated repeatedly to ead in order to allow the lysates to spread in an even manner. After the tissues were homogenized in an ice bath, the protein lysate was added for lysing at 4°C for 30 minutes, followed by periodic shaking at intervals of 10 minutes. The supernatants were obtained for further use after post‐centrifugation (12 000 rpm/min) at 4°C for 20 minutes and removal of lipid layer. The protein concentration of each sample was determined using a bicinchoninic acid (BCA) Kit (20201ES76, Shanghai Yeasen Biotechnology Co., Ltd., Shanghai, China), and the deionized water was used to ensure the consistency of the 30 μg sample loading. Stacking gel and 10% SDS running gel was prepared. The mixture of sample and loading buffer was boiled for at 100°C for 5 minutes. The proteins were then loaded onto an electrophoresis apparatus in each lane by micropipette after ice bath and centrifugation. The proteins were then transferred into nitrocellulose membranes. The membranes were blocked with 5% skim milk and incubated at 4°C overnight. The samples were incubated with rabbit anti‐S100A9 (ab105472, 1:1000), IL‐17 (ab79056, 0.5‐2 μg/mL), HMGB1 (ab79823, 1:10000), S100A12 (ab37657, 1:1000), TLR4 (ab83444, 1:1000) and RAGE (ab37647, 1:1000) primary antibodies overnight at 4°C on a shaking table. All aforementioned antibodies were purchased from Abcam Inc., Cambridge, MA, USA. Samples were washed 3 times with Tris‐buffered saline with Tween 20 (TBST, 5 minutes each time). The samples were subsequently incubated with goat anti‐rabbit IgG (FITC, 1:1000, Abcam Inc, Cambridge, MA, USA) secondary antibody at room temperature 1 hour. After 3 washes with TBST (5 minutes each time), chromogenic reagent was supplemented for developing. The Image J 1.48 software (National Institutes of Health, Bethesda, Maryland, USA) was used for quantitative analysis of proteins based on the ratio of grey value between proteins and GAPDH. The same procedure was conducted for all cell experiments after 48 hours of transfection.

### 2.8 Construction of lentiviral vectors

On the basis of the known mRNA sequence of S100A9 gene deposited in the GenBank database, siRNA design online software, BLOCK‐iT RNAi Designer (Invitrogen Inc., Carlsbad, CA, USA), was utilized to synthesize the primer sequences of shRNA1‐S100A9 and shRNA2‐S100A9 as well as the randomly selected NC sequences (Sigma, St. Louis, MO, USA) without targeting any gene. The sequences were as follows: shRNA1‐S100A9: Sense: 5′‐GCAGCATAACCACCATCATCG‐3′, Antisense: 5′‐CGATGATGGTGGTTATGCTGC‐3′; shRNA2‐S100A9: Sense: 5′‐GGACACAAACCAGGACAATCA‐3′, Antisense: 5′‐TGATTGTCCTGGTTTGTGTCC‐3′; Negative control: Sense: 5′‐GCGACGAUCUGCCUAAGAU‐3′, Antisense: 5′‐AUCUUAGGCAGAUCGUCGC‐3′. The synthesized single‐strand phosphorylation was annealed to form a double‐stranded DNA with double cleavage sites and cloned into lentiviral vector of pRNA‐Lenti‐GFPh. The recombinant plasmid expressing shRNA1 and shRNA2 were produced and transformed to *E‐coli* DH5α. A total of 16 single colonies were selected using medium containing ampicillin (A8180, AMRESCO, Inc., Solon, OH, USA) and amplified. The PCR amplification was then performed, followed by another preliminary selection. The plasmids were extracted using Gen Elute GenElute Plasmid Kit (PLD35‐1KT, Sigma, St. Louis, MO, USA) and further identified by DNA sequencing.

The 293T cells (ATCC‐Y0106, Shanghai Enzyme Research Biotechnology Co., Ltd, Shanghai, China) at the logarithmic growth phase were selected. After cell counting, the cells were inoculated with 5 × 10^6^ cells/culture dish in culture dishes and cultured in an incubator with 5% CO_2_ at 37°C overnight. After the removal of the former culture medium, a fresh serum‐containing medium was added to the cells. The virus solution was supplemented and mixed in its entirety in the cell suspension for incubation at 37°C. The cells were then added to a fresh medium with of the same volume after 4 hours to dilute the virus suspension, and cultured for 72 hours. A 5‐mL sterile centrifuge tube was prepared. Serum‐free Opti‐MEMI medium (40 μL) was inserted into the tube, with the subsequent supplementation of pLV/helper‐SL1, pLV/helper‐SL2, pHelper 2 (4 μL for each), followed by the upside down blending and incubation conducted under room temperature conditions for 5 minutes. Meanwhile, another 5‐mL sterile centrifuge tube was prepared, followed by the addition of serum‐free Opti‐MEMI medium as well as 40 μL lipofectamin 2000, and incubated for 5 minutes. The diluted lipofectamin 2000 was then added to the serum‐free medium containing Opti‐MEMI and mixed gently. After incubation at room temperature for 20 minutes, centrifugation was conducted at 3000 rpm for 15 minutes. Next, the supernatant was filtered with a 0.45‐μm filter to completely remove all cell debris. Precipitate in each tube was resuspended with 200 μL culture medium and then separately packed into 2 AXYGEN tubes (100 μL each tube) and stored at ‐80°C. The lentiviral titre was measured: Ten twofold serial dilutions of 100 μL lentivirus were added into 96‐well plates and cultured in an incubator containing 5% CO_2_ at 37°C for 24 hours. Three parallel plates were set for samples of each concentration. The dilution ratio with the highest fluorescence in lentivirus solution under fluorescence microscope observation was regarded as the lentiviral titre (unit IU/mL).

### 2.9 AP cell model establishment and grouping

The HPNE cells were purchased from ATCC (Maryland, US) and induced by caerulein to construct an AP cell model. The HPNE cells at the logarithmic growth phase were seeded into a 6‐well plate. After cell adhesion, the cells through the addition of 1 × 10^−8^ mol/L cerulein for 24 hours induced to establish an AP model. The cells were assigned into 5 groups: the control group (HPNE cells without transfection), blank group (HPNE cells induced by 1 × 10^−8^ mol/L cerulein without transfection), NC group (HPNE cells induced by 1 × 10^−8^ mol/L cerulein added with 1010 IU/mL shRNA‐S100A9 NC solution), shRNA1 group (HPNE cells induced by 1 × 10^−8^ mol/L cerulein added with 1010 IU/mL shRNA1‐S100A9 lentivirus solution) and shRNA2 group (HPNE cells induced by 1 × 10^−8 ^mol/L cerulein added with 1010 IU/mL shRNA2‐S100A9 lentivirus solution).

### 2.10 3‐(4,5‐dimethyl‐2‐thiazolyl)‐2,5‐diphenyl‐2‐H‐tetrazolium bromide (MTT) assay

At the 48 hours point, post‐infection with lentivirus, the cells were washed twice with PBS and digested with 0.25% trypsin for single cell suspension preparation. After the cells were counted, they were then inoculated in 96‐well plates (3 × 10^3^‐6 × 10^3^ cells/well) with 0.2 mL volume/well. Six reduplicate wells were set. The cells were incubated for 24, 48 and 72 hours, respectively, and continuously cultured for 4 hours in a medium containing 10% MTT solution (5 g/L, GD‐Y1317, Shanghai Guduo Biological Technology Co., Ltd., Shanghai, China). After removing the supernatant, dimethyl sulphoxide (DMSO, D5879‐100ML, Sigma, St. Louis, MO, USA) was added to each well (100 μL per well) and gently mixed for 5 minutes to completely dissolve the formazan crystals. The OD value was measured at a 590 nm using a microplate reader (BS‐1101, Nanjing DeTie Experimental Equipment Co., Ltd., Nanjing, China). All experiments were repeated 3 times. Cell viability curves were drawn with time‐point as abscissas and OD value as ordinates.

### 2.11 Flow cytometry

Propidium iodide (PI) staining was used to examine the cell cycle. At the 48 hours point post‐infection with lentivirus, the cells were collected and washed 3 times with ice‐cold PBS. After centrifugation, the supernatant was discarded. The cells were then re‐suspended in PBS and adjusted to a density of approximately 1 × 10^5^ cells/mL. The cells were then fixed with pre‐cooled 70% ice ethanol at ‐20°C and incubated at 4°C overnight. After centrifugation (800 g) at 4°C, the supernatant was discarded, and the cells were washed with PBS containing 1% foetal bovine serum (FBS). The cells were resuspended in 400 μL binding buffer. Next, the cells were incubated with 50 μL RNAase A (R4875, Shanghai Wegene Biotechnology Co., Ltd., Shanghai, China) at 37°C for 30 minutes. Then, 50 μL of 50 mg/L PI (GK3601‐50T, Beijing Dingguo Changsheng Biotechnology Co., Ltd., Beijing, China) was added in conditions void of light. The samples were once again washed with PBS and incubated at room temperature for 30 minutes. Finally, a flow cytometer was employed to analyse the cell cycle.

Annexin‐V‐fluorescein isothiocyanate (FITC)/PI double staining was used to evaluate cell apoptosis. At 48 h after transfection, the cells were digested with 0.25% trypsin without EDTA (YB15050057, Shanghai Yubo Biotechnology Co., Ltd., Shanghai, China), and collected to the flow tube. After centrifugation, the supernatant was discarded. The cells were then washed 3 times with ice‐cold PBS, and centrifuged, followed by the removal of the supernatant. In accordance with the instructions of Annexin‐V‐FITC Cell Apoptosis Detection Kit (K201‐100, BioVision, San Francisco, CA, USA), Annexin‐V‐FITC, PI and 4‐(2‐Hydroxyethyl)‐1‐piperazineethanesulfonic acid (HEPES) buffer with the ratio of 1:2:50 were mixed as Annexin‐V‐FITC/PI staining solution. The 1 × 10^6^ cells were resuspended with 100 μL staining solution. Next, the cells were shaken to permit mixing and incubated at room temperature for 15 minutes. The samples were added with 1 mL HEPES buffer (PB180325, Procell, Wuhan, China). At excitation of 488 nm, FITC fluorescence and PI fluorescence were measured by 515 and 620 nm bandpass filter, respectively, to evaluate cell apoptosis. The experiment was repeated 3 times.

### 2.12 Statistical analysis

All statistical analyses were performed using SPSS 21.0 software (International Business Machines Corporation (IBM) Company, New York, USA). Enumeration data were reported as rate or in percentage form. Comparisons among groups were analysed by chi‐square test. Measurement data were expressed as mean ± standard deviation (SD). The comparisons between two groups were analysed by means of *t* test, whereas comparisons among multiple groups were performed using one‐way analysis of variance (ANOVA). *P* < .05 was considered to be statistically significant.

## 3 RESULTS

### 3.1 Strong positive expressions of S100A9 and IL‐17 are found in pancreatic tissues

The expression of S100A9 determined by IHC displayed a weakly positive expression in the normal, AP + shRNA and AP + anti IL‐17 groups with light staining, but strongly positive expression in the AP, AP + NC and AP + IgG groups with a distinct increase in brown granules, of which were mainly expressed in the pancreatic ductal complex and interstitial inflammatory cells (Figure 1A). The positive expression of IL‐17 showed the same tendency with that of S100A9 (Figure 1B).

**Figure 1:** Positive expressions of S100A9 and IL‐17 in pancreatic tissues in each group determined by IHC. A, expression of S100A9 observed under the microscope (×400) and statistical analysis; B, expression of IL‐17 observed under the microscope (×400) and statistical analysis; *P <* *.05 compared with the normal group; ^#^ *P *<* *.05 compared with the AP group; S100A9, S100 calcium‐binding protein A9; IL‐17, interleukin 17; IHC, immunohistochemistry; AP, acute pancreatitis

### 3.2 S100A9 gene silencing attenuates pathological changes in pancreatic tissues

HE staining results exhibited that the pancreatic tissues in the normal group had clear structure, normal morphology without obvious bleeding or necrosis. There was obvious bleeding, vacuolization, focal necrosis and a large infiltration of neutrophils in the pancreatic and omental foci occurred in the AP, AP + NC and AP + IgG groups. But the AP + shRNA and AP + anti IL‐17 groups showed intact acini and lobules in pancreatic tissues, with no neutrophil infiltration except for mild oedema occurred in some interstitial areas (Figure 2).

**Figure 2:** Pathological morphology of pancreatic tissues in each group measured by HE staining (×200). HE, haematoxylin‐eosin

### 3.3 S100A9 gene silencing attenuates inflammatory response in AP mice

ELISA results revealed that when compared with the normal group, the expressions of AMY, LDH, CRP, TNFα, IL‐6 and IL‐8 in serum were significantly increased in the AP, AP + NC, AP + IgG, AP + shRNA and AP + anti IL‐17 groups (all *P *<* *.05). Compared with the AP, AP + NC and AP + IgG groups, the expressions of AMY, LDH, CRP, TNFα, IL‐6 and IL‐8 in serum were significantly decreased in the AP + shRNA and AP + anti IL‐17 groups (all *P *<* *.05). No significant differences were detected among the AP, AP + NC and AP + IgG groups (all *P *>* *.05; Table 2).

**Table 2:** Expressions of AMY, LDH, CRP, TNFα, IL‐6 and IL‐8 in serum in each group

Group	AMY (U/L)	LDH (U/L)	CRP (mg/L)	TNFα (pg/mL)	IL‐6 (pg/mL)	IL‐8 (pg/mL)
Normal	61.20 ± 7.32	410.25 ± 38.03	10.02 ± 2.56	24.05 ± 7.42	35.15 ± 8.51	9.25 ± 2.54
AP	283.03 ± 34.30^a^	982.30 ± 65.46^a^	46.21 ± 14.62^a^	51.12 ± 11.80^a^	67.58 ± 13.76^a^	38.69 ± 8.54^a^
AP + NC	289.28 ± 28.69^a^	975.26 ± 96.21^a^	48.73 ± 4.86^a^	49.51 ± 4.84^a^	64.17 ± 6.42^a^	40.26 ± 3.73^a^
AP + shRNA	153.28 ± 15.13^a^^,^ b	643.37 ± 60.25^a^^,^ b	29.63 ± 2.76^a^^,^ b	36.75 ± 3.22^a^^,^ b	51.28 ± 5.02^a^^,^ b	23.18 ± 2.13^a^^,^ b
AP + IgG	280.17 ± 28.36^a^	968.82 ± 9.69^a^	50.27 ± 5.01^a^	53.17 ± 5.42^a^	65.97 ± 6.42^a^	42.38 ± 4.16^a^
AP + anti IL‐17	159.37 ± 15.34^a^^,^ b	657.19 ± 62.35^a^^,^ b	27.37 ± 2.34^a^^,^ b	39.37 ± 3.76^a^^,^ b	48.73 ± 4.33^a^^,^ b	26.35 ± 2.34^a^^,^ b

AP, acute pancreatitis; NC, negative control; AMY, amylase; LDH, lactate dehydrogenase; CRP, c‐reactive protein; TNFα, tumour necrosis factor α; IL‐6, interleukin‐6; IL‐8, interleukin‐8.

a *P *<* *.05 compared with the normal group.

b *P *<* *.05 compared with the AP group.

### 3.4 S100A9 gene silencing blocks the activation of IL‐17 signalling pathway in vivo

Both RT‐qPCR and Western blotting indicated that the mRNA and protein expressions of S100A9, TLR4, RAGR, IL‐17, HMGB1 and S100A12 in the AP group were all higher than those in the normal group (all *P *<* *.05). The AP + shRNA group had significantly lower mRNA and protein expressions of S100A9, TLR4, RAGR and HMGB1, as well as an insignificant reduction in the expressions of IL‐17 and S100A12 compared with the normal group. Furthermore, there were significantly lower mRNA and protein expressions of S100A9, TLR4, RAGR, IL‐17 and HMGB1, while insignificant reductions in the expressions of S100A12 in the AP + anti IL‐17 group. There was no significant difference detected among the AP, AP + NC and AP + IgG groups (*P *>* *.05; Figure 3A, B).

**Figure 3:** Relative mRNA and protein expressions of S100A9, TLR4, RAGE, IL‐17, HMGB1 and S100A12 in pancreatic tissues in each group examined by RT‐qPCR and Western blotting. (A) mRNA expressions of S100A9, TLR4, RAGE, IL‐17, HMGB1 and S100A12 in pancreatic tissues in each group examined by RT‐qPCR; (B) protein expressions of S100A9, TLR4, RAGE, IL‐17, HMGB1 and S100A12 in pancreatic tissues in each group examined by Western blotting; *P <* *.05 compared with the normal group; ^#^ *P *<* *.05 compared with the AP group; S100A9, S100 calcium‐binding protein A9; TLR4, toll‐like receptor 4; RAGE, receptor for advanced glycation end products; IL‐17, interleukin‐17; HMGB1, high‐mobility group box 1 protein; S100A12, calgranulin (C) RT‐qPCR, reverse transcription quantitative polymerase chain reaction; AP, acute pancreatitis

### 3.5 S100A9 gene silencing blocks the activation of IL‐17 signalling pathway in vitro

In comparison with the control group, the blank, NC, shRNA1 and shRNA2 groups had increased mRNA and protein expressions of S100A9, TLR4, RAGE, IL‐17, HMGB1 and S100A12 (all *P *<* *.05). Compared with the blank and NC groups, the shRNA1 and shRNA2 groups had displayed notably decreased mRNA and protein expression of S100A9, TLR4, RAGE and HMGB1, as well as no significant declines in the expressions of IL‐17 and S100A12. No significant difference was observed between the shRNA1 and shRNA2 groups (Figure 4; *P *>* *.05).

**Figure 4:** Relative mRNA and protein expressions of S100A9, TLR4, RAGE, IL‐17, HMGB1 and S100A12 in HPNE cells in each group determined by RT‐qPCR and Western blotting. (A) protein expressions of S100A9, TLR4, RAGE, IL‐17, HMGB1 and S100A12 in HPNE cells in each group determined by Western blotting; (B) mRNA expressions of S100A9, TLR4, RAGE, IL‐17, HMGB1 and S100A12 in HPNE cells in each group determined by RT‐qPCR; *P <* *.05 compared with the control group; ^#^ *P *<* *.05 compared with the blank and NC group; S100A9, S100 calcium‐binding protein A9; TLR4, toll‐like receptor 4; RAGE, receptor for advanced glycation end products; IL‐17, interleukin‐17; HMGB1, high‐mobility group box 1 protein; S100A12, calgranulin (C) RT‐qPCR, reverse transcription quantitative polymerase chain reaction; GAPDH, glyceraldehyde‐3‐phosphate dehydrogenase; AP, acute pancreatitis

### 3.6 S100A9 gene silencing increases cell proliferation

Compared with the control group, cell proliferation in the blank, NC, shRNA1 and shRNA2 groups was reduced, when measured after 48 and 72 hours (all *P *<* *.05). However, no significant difference was found between the blank and NC groups at each point (all *P *>* *.05). Compared with the blank and NC groups, the shRNA1 and shRNA2 groups showed increased proliferation capacities both at 48 and 72 hours, whereas the proliferation capacities of the shRNA1 group were slightly higher than that in the shRNA2 group (*P > *.05; Figure 5).

**Figure 5:** Cell proliferation in each group evaluated by MTT assay. *P <* *.05 compared with the control group; ^#^ *P *<* *.05 compared with the blank and NC groups; NC, negative control; OD, optical density; MTT, 3‐(4,5‐dimethyl‐2‐thiazolyl)‐2,5‐diphenyl‐2‐H‐tetrazolium bromide

### 3.7 S100A9 gene silencing promotes cell cycle entry while decreasing cell apoptosis

PI staining results illustrated in Figure 6A and B indicated that when compared with the control group, the percentage of cells at the G1 phase had increased, whereas reductions at the G2 and S phases were recorded in the blank, NC, shRNA1 and shRNA2 groups (all *P *<* *.05). There were no statistically significant differences observed between the blank and NC groups (all *P *>* *.05). Compared with the blank and NC groups, the percentage of cells decreased at the G1 phase; however, increases at G2 and S phases in the shRNA1 and shRNA2 groups were observed (all *P *<* *.05). Among cells in the shRNA1 group decreases of cells at the G1 phase but increases at G2 and S phase in comparison with the shRNA2 group were observed.

**Figure 6:** Cell cycle distribution and cell apoptosis measured by flow cytometry A and B, cell cycle distribution in each group; C and D, cell apoptosis rate in each group; *P <* *.05 compared with the control group; ^#^ *P *<* *.05 compared with the blank and NC groups; NC, negative control

Annexin‐V‐FITC/PI double‐staining results shown in Figure 6C and D revealed that comparisons of the apoptotic rate in the control group (5.26 ± 0.53)% revealed increased apoptotic rates in the blank group (18.36 ± 1.86)%, the NC group (19.23 ± 1.92)%, the shRNA1 group (11.36 ± 1.16)% and the shRNA2 group (12.01 ± 1.20)% (all *P *<* *.05). No significant difference was found between the blank and NC groups (*P *>* *.05). Compared with the blank and NC groups, the shRNA1 and shRNA2 groups had decreases in apoptotic rates (all *P *<* *.05). The apoptotic rate in the shRNA1 group was slightly lower than that in the shRNA2 group (*P *>* *.05).

## 4 DISCUSSION

The prognosis of AP is generally unfavourable, whereas the rate of recurrence is as high as 17%. Approximately 8% of AP patients will fall victim to chronic pancreatitis within a 5‐year period.^20^ Therefore, it is of significant urgency that more effective treatments are used to alleviate the issue of recurrence. Our findings provided evidence that S100A9 silencing inhibited the release of inflammatory cytokines, suppressed the proliferation and promoted apoptosis of pancreatic cells in a mouse model of AP, via the blockade of the IL‐17 signalling pathway, thus highlighting the potential of S100A9 as a therapy target in the treatment of AP.

Elevated expression of S100A9 has previously been detected in the progression of a number of inflammatory diseases, including psoriatic arthritis,^21^ systemic lupus erythematosus^22^ and inflammatory bowel disease.^23^ Likewise, this was detected in our results, in which we identified increased expression of S100A9 in our AP mice models. As a member of the S100 family, with the exception of those affecting epithelial tissues, S100A9 maintains its regulatory influence on cellular processes including transcription, proliferation and differentiation.^24^ In addition, combined with its heterodimer partner S100A8, S100A9 exerted growth‐inhibitory and apoptosis‐inducing effects in a variety of cells via the classical mitochondrial pathway.^25^, ^26^ Moreover, Li et al asserted that the overexpression of S100A9 could induce cell apoptosis and inhibit cell growth.^27^ Therefore, during our study, it was inferred that S100A9 gene silencing could act to promote cell growth and inhibit cell apoptosis in AP. S100A8/S100A9 was shown to control the G2/M cell cycle checkpoint as well as the apparent dysregulation that occurred, leading to the loss of the checkpoint in head and neck squamous cell carcinoma.^28^ During the process, p53, correlated with cell cycle, apoptosis and adipogenesis, can modulate S100A9 transcription.^29^ Initially, S100A8/A9 enhanced the activity of PP2A phosphatase as well as p‐Chk1 (Ser345) phosphorylation, leading to the inactivation of the G2/M Cdc2/cyclin B1 complex through the inhibitory phosphorylation of mitotic p‐Cdc25C (Ser216) and p‐Cdc2 (Thr14/Tyr15); followed by the decrease in the expression of Cyclin B1 and cell cycle arrest at the G2/M checkpoint, which ultimately resulted in the reduction in cell division and the negative regulation squamous cell carcinoma growth.^30^ In a zinc‐reversible manner, S100A8/A9 induced apoptosis in various human and mouse tumour cell lines, including colon cancer cell lines.^31^ In a previous study reported by Schnekenburger et al, he and his team found that pancreatitis induced an increased level of S100A9 in the pancreas and the application of S100A8/A9 in mice induces pancreatic cell‐cell contract dissociation which could trigger cell apoptosis.^32^ Once the activation of the IL‐17 signalling pathway is mediated by S100A9, HMGB1 and RAGE both of which are cell death biomarkers are up‐regulated, thus leading to cell apoptosis.^33^

IL‐17 is characterized by its ability to induce the expression of both cytokines and chemokines and has been reported to participate in the amplification of inflammatory responses.^34^ The significant effects of IL‐17 blockade have proved to be controversial, due to its weak functions in vitro, as on the one hand IL‐6 secretin, nuclear factor‐κB (NF‐κB) or other pro‐inflammatory, which were only activated under high levels of cytokines, whereas on the other hand IL‐17 exhibited significantly potent synergy in its ability to link with other cytokines such as IL‐1β and TNFα.^35^ In the present study, we found that S100A9 exerted its effects by blocking the IL‐17 signalling pathway. This was supported by a study reviewing the synovial fluid (SF) of rheumatoid arthritis (RA), which initially indicated that S100A9 level was closely associated with IL‐17 and IL‐6, the critical factor to induce T‐helper (Th) 17 differentiations.^36^ Meanwhile, the activation of Th17 cells resulted in the production of IL‐17 expression and overexpression of IL‐17, together with TNF, may lead to cartilage surface erosion.^37^ A clinical study reported by Jia et al demonstrated that the serum level of IL‐17 might be linked to AP severity and sever as a prognostic factor in evaluating disease severity of patients with AP.^38^

S100A8 and S100A9 are generally considered to be pro‐inflammatory substances.^39^ This was observed in the present study in that S100A9 silencing inhibited the release of pro‐inflammatory cytokines. Both the pro‐ and anti‐inflammatory functions of macrophages were primarily premised on the following factors: One was the stage of differentiation and the other was distinct mechanisms of activation.^40^ Considering that S100A8 and S100A9 were less stable than S100A8/A9 heterodimers, S100A8/A9 heterodimers are usually referred to when discussing pro‐inflammatory activities.^41^ The main receptors for S100A8, S100A9 and calprotectin are TLR4, which represent the dominant receptor for the S100A8/S100A9 signalling pathway, as well as RAGE; however, the specific receptors and pathways for S100A8, S100A9 and calprotectin are mainly dependent on the cell type.^42^ For example, activated microglia produces significantly greater levels of S100A9 in Alzheimer's disease.^43^ A previous study indicated that both TLR4 and RAGE proteins were overexpressed in pancreatitis, as well as highlighting the ability of S100A9 to activate the IL‐17 signalling pathway and regulate the expression of inflammatory factors by binding to the cell surface receptors TLR4 and RAGE proteins.^44^ Once secreted, S100A8/S100A9 has the potential to bind to TLR4, which displayed pro‐inflammatory functions, and result in the up‐regulation of pro‐inflammatory cytokines, the activation of endothelial cells and macrophages.^36^

In conclusion, the results of the present study demonstrated that S100A9 silencing inhibits the release of pro‐inflammatory cytokines by blocking the IL‐17 signalling pathway. This was evidentiary the established AP mouse model in this study. Cell proliferation was inhibited, and apoptosis conditions were enhanced. The results of this study provide an experimental basis for the use of S100A9‐based therapy in the treatment of AP. It should be noted that the mechanisms between S100A9 and the IL‐17 signalling pathway require further analysis and further clinical trials are needed, in order to assess whether the key findings of this study can be applied to human beings.

## CONFLICT OF INTEREST

None.
